The article "The long non‐coding RNA‐ROR promotes osteosarcoma progression by targeting miR‐206" was retracted in 2024. Reasons: duplicated images; unreliable results or conclusions.

# The long non‐coding RNA‐ROR promotes osteosarcoma progression by targeting miR‐206

**DOI:** 10.1111/jcmm.14087

**Published:** 2018-12-19

**Authors:** Dan Fei, Guoqing Sui, Yang Lu, Long Tan, Zhao Dongxu, Kewei Zhang

**Affiliations:** ^1^ Ultrasonographic Department China‐Japan Union Hospital of Jilin University Changchun P.R. China; ^2^ Department of Orthopaedic Surgery China‐Japan Union Hospital of Jilin University Changchun P.R. China; ^3^ Department of Thoracic Surgery The First Hospital of Jilin University Changchun P.R. China

**Keywords:** invasion, lncRNA, miR‐206, osteosarcoma, proliferation, ROR

## Abstract

The long intergenic non‐protein coding RNA regulator of reprogramming (lncRNA‐ROR) has been reported to play crucial regulatory roles in the pathogenesis and progression of multiple cancers. However, whether ROR is associated with the initiation and development of osteosarcoma (OS) remains unclear. Here, we found that ROR expression level was significantly up‐regulated in OS tissue samples compared to adjacent normal tissues, and the elevated ROR was closely correlated with advanced tumour‐node‐metastasis (TNM) stage and lymph node metastasis and poor overall survival rate. Functional assays showed that ROR knockdown suppressed the OS cell proliferation, colony formation, migration and invasion in vitro, and retarded tumour growth in vivo. In addition, miR‐206 was verified to be a target miRNA of ROR using bioinformatics online program and luciferase report assay. miR‐206 inhibition partially rescued the inhibitory effects on OS cells induced by ROR knockdown. In conclusion, these results suggested that ROR function as an oncogene in OS by sponging miR‐206 and might be a potential therapeutic target for patients with OS.

## 1 INTRODUCTION

Osteosarcoma (OS), stemming from bone‐forming mesenchymal cell, is a primary malignant bone tumour for children and adolescents.^1^ Despite great progression has been made in early diagnosis and combination treatment of human OS, the prognosis of patients, especially with recurrent and metastatic sarcomas, still remains poor.^2^ Therefore, it is urgent need to understand the molecular mechanism of OS carcinogenesis to unearth reliable diagnostic and therapeutic targets for the treatment of this disease.

Long non‐coding RNAs (lncRNAs) are a family of over 200‐nucleotide RNA molecules in length without protein‐coding capacity.^3^ Long non‐coding RNAs have been reported to be involved in regulating various biological procession, such as cell proliferation, apoptosis, differentiation and invasion.^4^, ^5^ Recently, a number of lncRNAs have been demonstrated to be abnormally expressed in various cancers, and play crucial roles in initiation and development of various cancers^.^ 6, 7 Many lncRNAs were identified to implicate in regulating OS pathogenesis such as cell growth, apoptosis and metastasis, suggesting that lncRNA could serve as a diagnosis marker and therapy target for OS.^8^, ^9^

Recently, long intergenic non‐protein coding RNA, regulator of reprogramming (lncRNA‐ROR) was found to be up‐regulated, and function as oncogene in non‐small lung cancer,^10^ breast cancer,^11^ renal cancer,^12^ prostate cancer,^13^ esophageal squamous cell carcinoma^14^ and hepatocelluar carcinoma.^15^ However, its potential prognostic value and biological function in OS have not yet been explored. In our study, we tried to study the prognostic value and biological function of ROR in OS. Our data revealed that ROR expression was up‐regulated in OS tissues and cell lines. ROR knockdown significantly inhibited OS cell proliferation, colony formation, migration and invasion by partially regulating the miR‐206. These findings suggested that ROR might be a potential target for the diagnosis and treatment of OS.

## 2 MATERIALS AND METHODS

### 2.1 Tissue samples

The human OS tissues (OS) and the adjacent normal bone tissues (ANT) were obtained from 48 OS patients who received surgical treatment at China‐Japan Union Hospital of Jilin University (Changchun, China). None of patients received chemotherapy or radiotherapy prior to surgery. All tissues were immediately frozen and stored in liquid nitrogen for further analysis. The use of human tissues was approved by the author hospital's ethics committees. All patients or their family members signed a written consent form. Clinical and pathological data were acquired from the medical records, and listed in Table1.

**Table 1:** Correlation between clinicopathological features and regulator of reprogramming (ROR) expression in 48 patients with osteosarcoma

Variables	No. of cases	ROR expression		*P* value
		High (n %)	Low (n %)	
Age (y)				*P* > 0.05
<20	28	16 (57.1)	12 (42.9)	
≥20	20	10 (50.0)	10 (50.0)	
Gender				*P* > 0.05
Male	25	14 (56.0)	11 (44.0)	
Female	23	12 (52.2)	11 (47.8)	
TNM stage				*P* < 0.01
I‐II	37	16 (43.2)	21 (56.8)	
III‐IV	11	10 (90.9)	1 (9.1)	
Tumour size				*P* > 0.05
<3 cm	30	16 (53.3)	14 (46.7)	
≥3 cm	18	10 (55.6)	8 (44.4)	
Metastasis				*P* < 0.01
No	38	16 (42.1)	16 (57.9)	
Yes	10	10 (100)	0 (0)	

TNM, tumour‐node‐metastasis.

### 2.2 Cell culture

The established human OS cell lines including Saos‐2, U2OS, MG‐63 and 143B and normal human osteoblasts, hFOB 1.19, were purchased from American Type Culture Collection (Manassas, USA), were maintained in Dulbecco's modified Eagle's medium (DMEM; Gibco, CA, USA) containing with 10% foetal bovine serum (FBS, Gibco) and 100 units/mL of penicillin and streptomycin (Invitrogen, CA, USA) in a humidified 5% CO_2_ incubator at 37°C.

### 2.3 Transfection and generation of stably transfected cell lines

Two different sequences of short‐hairpin RNA (shRNA) against ROR were designed and synthesized by GenePharma (Shanghai, China) and was transfected into U2OS cells, and were respectively referred as to sh‐ROR#1 and sh‐ROR#2. For overexpressing or suppressing the expression of miR‐206, miR‐206 mimic, mimic negative control (miR‐NC) and miR‐206 inhibitor were synthesized by Ribobio (Guangzhou, China) and were respectively transfected into U2OS cells using Lipofectamine 2000 (Invitrogen) according to the manufacturer's protocols. The stably transfected cells were selected by 0.5 mg/mL G418 (Sigma‐Aldrich) at 48 hours of transfection. At about 28 days, stable cells (G418‐resistant cell clones) were established.

### 2.4 Real‐time RT‐PCR

Total RNA was extracted from tissue samples and cultured cells using TRIzol^®^ reagent (Invitrogen; Thermo Fisher Scientific, Inc.) according to the manufacturer's protocol. The relative expression of miR‐206 was examined using a SYBR PrimeScript miRNA RT PCR kit (Takara, Dalian, China) on an Applied Biosystems 7900 Sequence Detection system (Applied Biosystems, Foster City, CA, USA) using specific primer (Applied Biosystems). U6 was used as an internal control. For detection of ROR expression, RNA samples were reverse‐transcribed into cDNA by using PrimeScript^®^ RT Master Mix Perfect Real‐Time (Takara), then was quantified using SYBR Geen Master Mix (Applied Biosystems) on an Applied Biosystems 7900 Sequence Detection system. Primers used in this study were as follows: ROR forward 5′‐CTTGATGGCATTGTCGCTAA‐3′, reverse 5′‐TCCAGTGGCTGTGCTAGATG‐3′; GAPDH forward 5′‐TCGGAGTCAACGGATTTGGT‐3′, reverse 5′‐TTGGAGGGATCTCGCTCCT‐3′. GAPDH was used as an internal control. The relative expression miRNA or mRNA was determined using the $2^{-\Delta \Delta C_{t}}$ method.

### 2.5 Cell proliferation assay

Cell viability was detected using Cell Counting Kit‐8 (CCK‐8; Dojindo Molecular Technologies, Inc., Kumamoto, Japan). Briefly, transfected cells were seeded into 96‐well plates at a density of 5,000 per well. At different time‐points (24, 48 and 72 hours), 10 μL CCK‐8 solution was added in each well and additionally for 4 hours at 37°C. Absorbance was measured at a wavelength of 450 nm for each sample by a microplate reader (Bio‐Rad, Hercules, CA, USA).

### 2.6 Colony formation assay

For the colony formation assay, stable ROR‐depletion cells grown in 6‐well plates (in triplicate), and allowed to adhere and cultured for 10 days. Then cell colonies were fixed with 96% ethanol for 10 minutes and stained with 1% crystal violet for 5 minutes. The colonies were imaged and counted using an inverted microscope (Olympus Corporation, Tokyo, Japan).

### 2.7 Migration and invasion assays

Cell migration was determined by a wound‐healing assay. Briefly, transfected cells were cultured in 6‐well plates (5 × 10^4^ cells per well) and grown to 100% confluence. Subsequently, an artificial homogenous wound was created in the monolayer using a sterile plastic micropipette tip, and cultured for 24 hours in serum‐free medium. Photographs were taken 0 and 24 hours after wound using an X71 inverted microscope (Olympus). The wound areas were analysed by Image j software (National Institutes of Health, Bethesda, MD, USA).

Cell invasion was examined using Matrigel invasion assays. Briefly, 1 × 10^5^ transfected cells in 100 uL free‐serum DMEM medium were seeded into the upper chamber of Transwell chamber pre‐coated with 100 mL of Matrigel (BD Biosciences, San Jose, CA, USA), while DMEM medium supplemented with 20% FBS was added to the lower chamber. After incubation for 24 hours at 37°C in a 5% CO_2_ atmosphere, the non‐invading cells were removed using cotton swab; the invading cells were fixed with 4% paraformaldehyde for 15 minutes and stained with 1% crystal violet for 30 minutes at 37°C. Invasive cells were counted in five randomly selected fields and observed under a light microscope (Olympus Corporation).

### 2.8 Bioinformatics, miRNA‐target identification and luciferase assay

A target prediction tool RNA 22 was used to predict potential ROR targets. A luciferase assay was performed to validate prediction of binding sites between ROR and miR‐206. Briefly, the 3′ untranslated region (UTR) of ROR containing a potential binding site for miR‐206 was synthesized and inserted into a luciferase‐reporter vector psiCHECK2 (Promega Corporation, Madison, WI, USA) and designated as ROR wild‐type (Wt). A mutant (Mut) version of the ROR 3′ UTR was constructed using the QuikChange XL site‐directed mutagenesis kit (Agilent Technologies, Santa Clara, CA, USA) according to the manufacturer's protocol, and referred as ROR Mut. For the luciferase assay, U2OS cells were grown to 70%‐80% confluence in 24‐well plates and cotransfected with a miR‐206 mimic or miR‐NC and ROR Wt or ROR Mut reporter plasmids using Lipofectamine 2000 (Invitrogen) following the manufacturer protocol. Firefly luciferase and Renilla luciferase were determined using a dual‐luciferase reporter assay (Promega Corporation) at 48 hours after transfection following the manufacturer's protocol, and Renilla luciferase activity was normalized against that of firefly luciferase.

### 2.9 Tumour xenograft model

All animal experiments were reviewed and approved by the Institutional Animal Care and Use Committee of the Jilin University (Changchun, China). Male athymic BALB/c nude mice (4‐5 weeks old, 18‐20 g) were brought from the Experimental Animal Center of Changchun (Changchun, China), and were maintained in specific pathogen‐free conditions.

U2OS cells (2 × 10^6^) stably transfected with sh‐ROR or sh‐NC were subcutaneously injected into the flanks of nude mice respectively. The tumour volume (V) was monitored every 7 days until the mice were killed. The tumour volume was calculated following the formula: V = 0.5 × (L × W^2^) by measuring tumour length (L) and width (W). At 4 weeks after injection, the mice were killed, and the tumours were carefully stripped, photographed, weighed and stored in liquid nitrogen for further experiments.

### 2.10 Immunohistochemistry staining

Immunohistochemistry (IHC) was conducted by previously described methods.^16^, ^17^ Sections of tissues were incubated with antibodies against Ki‐67 (1:100 dilution; D2H10, CST, Danvers, USA).

### 2.11 Statistical analysis

All experiments were conducted at least three times. The data shown in this study were presented as mean ± SD. Statistical analysis was made by utilizing the spss 17.0 software (spss Inc., Chicago, IL, USA) and GraphPad Prism 5.0 software (GraphPad Software Inc., La Jolla, CA, USA). Two groups of comparisons were carried out with a Student's *t* test. Multiple comparisons were performed with one‐way ANOVA. Correlations between ROR expression and miR‐206 expression were evaluated by Pearson's correlation analysis. Log‐rank test was used for Kaplan‐Meier survival curve analysis. A *P* value <0.05 or less was considered as statistically significant.

## 3 RESULTS

### 3.1 ROR is up‐regulated in OS tissues and cell lines

ROR expression in 48 paired OS tissues and corresponding adjacent non‐tumour tissues was examined by real‐time quantitative PCR (qRT‐PCR), revealing that OS tissues exhibited higher ROR expression compared with ANT (Figure 1A). It was also revealed that increased ROR was positively associated with advanced TNM stage and lymph node metastasis (Table1). Osteosarcoma patients were further divided into two subgroups based on mean of ROR expression. Shorter overall survival was observed in OS patients with high ROR expression than those with low ROR expression level (Figure 1B). ROR expression in four OS cell lines Saos‐2, U2OS, MG‐63 and 143B was examined, and qRT‐PCR results revealed that ROR levels in four human OS cell lines were significantly up‐regulated compared with normal human osteoblasts, hFOB 1.19 (Figure 1C). These data suggested that ROR might be involved in OS carcinogenesis.

**Figure 1:** Regulator of reprogramming (ROR) was up‐regulated in osteosarcoma (OS) tissues and cell lines. (A) qRT‐PCR analysed the level of ROR in OS tissues and adjacent normal tissues (n = 48). (B) Kaplan‐Meier survival curve and log‐rank test were used to evaluate the correlation between the expression of ROR and overall survival of patients with OS. (C) qRT‐PCR analysed the level of ROR in OS cell lines (Saos‐2, U2OS, MG‐63 and 143B) and normal human osteoblasts, hFOB 1.19. **P < 0.01

### 3.2 ROR knockdown inhibits OS cell proliferation and colony formation

To determine the effects of ROR on cell proliferation in OS, ROR was knocked down in U2OS cells by transfection with sh‐ROR1# and sh‐ROR2#. We found that U2OS cells transfected with sh‐ROR1# and sh‐ROR2# significantly decreased ROR expression compared to cells transfected with sh‐NC (Figure 2A). sh‐ROR1# exhibited greater effect on expression of ROR in U2OS, which showed a 75.8% decrease, as confirmed at transcriptional levels (Figure 2A). Therefore, sh‐ROR1# was chosen as a candidate shRNA for all subsequently studies, and was designated as sh‐ROR. CCK‐8 assay demonstrated that SOR knockdown in U2OS cells significantly decreased proliferation (Figure 2B). Consistent with these results, ROR knockdown significantly decreased colony formation of U2OS cells (Figure 2C).

**Figure 2:** Knockdown of regulator of reprogramming (ROR) inhibited osteosarcoma (OS) proliferation and colony formation. (A) qRT‐PCR analysed the level of ROR in U2OS cells transfected with Sh‐ROR#1, sh‐ROR#2 or si‐NC. (B) CCK8 assay was used to evaluate the effect of ROR knockdown on U2OS cell proliferation. (C) Colony formation assay was employed to evaluate the effect of ROR knockdown on U2OS cell colony formation. *P < 0.05, **P < 0.01

### 3.3 ROR knockdown inhibits OS cell migration and invasion

The effects of ROR knockdown on cell migration and invasion in OS cells were determined by wound healing assay and transwell invasion assay respectively. The wound healing assay showed that ROR knockdown in U2OS cells attenuated the cell migration abilities (Figure 3A). The transwell invasion assay demonstrated that knockdown of ROR in U2OS cells caused a significant decrease in the number of invaded cells (Figure 3B).

**Figure 3:** Knockdown of regulator of reprogramming (ROR) inhibited osteosarcoma (OS) migration and invasion. (A) Wound healing assay was employed to investigate the effect of ROR knockdown on U2OS cell migratory capacity. (B) Transwell invasion assay was employed to evaluate the effect of ROR knockdown on U2OS cell invasive capacity. **P < 0.01

### 3.4 miR‐206 was a target of ROR in OS

To explore the potential mechanisms of ROR functions in OS cells, a target prediction tool RNA 22 was employed to search the potential targets of ROR. Bioinformatic tool analysis demonstrated a potential binding site for miR‐206 on ROR gene (Figure 4A). The luciferase reporter assays further manifested that miR‐206 overexpression significantly suppressed the luciferase activity that carried Wt but not Mut 3ʹ‐UTR of ROR in U2OS cells (*P* < 0.05, Figure 4B). Moreover, the qRT‐PCR data revealed that miR‐206 overexpression significantly suppressed ROR expression in U2OS cells (Figure 4C), while ROR silencing resulted in an increased expression of miR‐206 in U2OS cells (Figure 4D). We also demonstrated that the expression of miR‐206 was markedly down‐regulated in OS tissues compared to adjacent normal tissues (*P* < 0.01, Figure 4E). Pearson correlation analysis revealed that miR‐206 expression was negatively correlated with ROR expression in OS tissues (*r* = −0.576, *P < *0.001, Figure 4F). Combined with the findings above, we believed that miR‐206 was a target of ROR in OS cells.

**Figure 4:** miR‐206 was a target of regulator of reprogramming (ROR) in osteosarcoma (OS) cells. (A) Binding and mutant sites between miR‐206 and ROR. (B) Luciferase activity was detected in U2OS cells after cotransfection with miR‐206 mimic/miR‐NC mimic and ROR Wt or ROR Mut reported plasmid. (C) The expression of ROR in U2OS cells transfected with miR‐206 mimic or sh‐NC. (D) The expression of miR‐206 in U2OS cells transfected with Sh‐ROR or Sh‐NC. (E) The expression of miR‐206 in OS tissues and adjacent normal tissues (n = 48). (F) Correlation between ROR expression and miR‐206 expression in OS tissues was analysed by Pearson's correlation analysis.**P < 0.01

### 3.5 ROR knockdown inhibits OS cell progression via up‐regulation of miR‐206

Next, the effects of miR‐206 on ROR‐modulated cell proliferation, colony formation, migration and invasion of U2OS cells were investigated. We knocked down ROR and inhibited miR‐206 at the same time in U2OS cells(Figure 5A), after which cell proliferation, colony formation, migration, invasion of U2OS cells were determined by CCK8, colony formation, wound healing and transwell invasion assays respectively. Results identified that ROR knockdown inhibited cell proliferation, colony formation, migration and invasion of U2OS cells, and the inhibitory effects were attenuated when miR‐206 was down‐regulated (all *P* < 0.05, Figure 5B‐E).These data suggested that ROR knockdown inhibited OS progression via up‐regulation of miR‐206.

**Figure 5:** miR‐206 inhibitor rescued the inhibitory effect on proliferation, colony formation, migration and invasion of osteosarcoma (OS) cells induced by regulator of reprogramming (ROR) depletion. (A) The expression of miR‐206 was examined in U2OS cells transfected with Sh‐NC, Sh‐ROR and Sh‐ROR+miR‐206 inhibitor. (B‐E). Cell proliferation, colony formation, migration and invasion were detected in U2OS cells transfected with Sh‐NC, Sh‐ROR and Sh‐ROR+miR‐206 inhibitor. *P < 0.05, **P < 0.01

### 3.6 ROR knockdown inhibits tumour growth in vivo

To explore whether ROR could also regulate tumourigenesis in vivo, we performed a xenograft tumour growth assay. The U2OS cells stable transfected with sh‐ROR and sh‐NC respectively were injected into nude mice, and tumour growth was determined. We observed that xenograft tumour growth was slower in sh‐ROR injection group than that of sh‐NC group (Figure 6A). At 28 days post‐injection, the mice were killed and tumour tissues were stripped and weighted. Average tumour size and weight were significantly decreased in sh‐ROR injection group compared to sh‐NC injection group (Figure 6B,C). In addition, IHC assay demonstrated that the proliferation marker Ki‐67 expression was significantly decreased in the sh‐ROR injection group compared to sh‐NC group (Figure 6D). Finally, our results revealed that ROR expression was down‐regualted in sh‐ROR injection group (Figure 6E), while miR‐206 expression was up‐regulated in sh‐ROR injection group (Figure 6F). These results suggested that the knockdown of ROR suppresses tumour growth in vivo.

**Figure 6:** Regulator of reprogramming (ROR) knockdown inhibits tumour growth in vivo. (A) The tumour growth curves of nude mice were established (B) The tumour image. (C)The tumour’s weight. (D) The Ki‐67 expression was determined in xenograft tumour by IHC. (E) qRT‐PCR analysed the level of ROR in xenograft tumour. (F) qRT‐PCR analysed the level of miR‐206 in xenograft tumour. **P < 0.01

## 4 DISCUSSION

Nowadays, accumulating evidence demonstrated that dysregulation of lncRNAs had crucial functions in growth and metastasis of various types of cancer.^18^, ^19^ More and more LncRNAs have been confirmed to be involved in progression and development of OS.^20^ For example, Gu et  al reported that LINC00858 significantly promoted OS cells' proliferation and invasion in vitro, and increased tumour growth in vivo through regulating miR‐139‐CDK14 axis.^21^ Xie et  al reported that lncRNA TUG1 promoted cell proliferation and suppressed apoptosis in OS cells by regulating miR‐212‐3p/FOXA1 axis.^22^ Yang et  al demonstrated that knockdown of lncRNA TP73‐AS1 inhibited OS cell proliferation and invasion through sponging miR‐142.^23^ Here, we found that knockdown of ROR inhibited OS progression by regulating miR‐206, which provides a new molecular target for the treatment of OS.

Long non‐coding RNA‐ROR, a newly‐discovered non‐coding RNA, was first reportedly to act as a p53 repressor in response to DNA damage.^24^ Accumulating evidence showed that ROR implicated in the initiation and development of various cancers.^10^, ^11^, ^12^, ^13^, ^14^, ^15^ However, the specific effect of ROR on the occurrence and progression of OS remains unclear. Here, ROR was found to be strongly expressed in OS tissues and cell lines. Higher ROR was positively related to advanced TNM stage and lymph node metastasis and poor overall survival. Functional assay demonstrated that knockdown of ROR significantly inhibited the proliferation, colony formation, migration and invasion of OS cells, as well as suppressed tumour growth in vivo. Those results implicated that ROR functions as an oncogene in OS.

Long non‐coding RNAs were reported to exert their biological roles by functioning as competing endogenous RNAs (ceRNAs) to negatively regulate the miRNA expressions.^25^ To investigate the underlying mechanisms by which ROR exerts its biological effects on OS cell proliferation and invasion, it is necessary to identify its binding miRNAs. A bioinformatics tool (RNA22) was employed to search the potential target of ROR. Among target miRNAs, miR‐206 was chosen as a candidate miRNA for further investigation based on its biological function in OS.^26^, ^27^, ^28^ miR‐206 has been reported to function as the tumour suppressor miRNA in multiple cancers, such as ovarian cancer,^29^ non‐small lung cancer,^30^ cervical cancer,^31^ gastric cancer^32^ and colorectal cancer.^33^ Previous studies demonstrated that miR‐206 expression was down‐regulated in OS tissues and cell lines, and that overexpression of miR‐206 inhibits OS cell proliferation, migration and invasion by targeting multiple genes.^26^, ^27^, ^28^ Although recently a study showed that ROR promoted esophageal squamous cell carcinoma progression via sponging multiple miRNAs including miR‐206,^14^ the association with miR‐206 and ROR in OS remained unclear. In the present study, miR‐206 was identified as a downstream target of ROR by luciferase‐reporter assay. miR‐206 overexpression significantly suppressed ROR expression in U2OS cells, while ROR silencing resulted in an increased expression of miR‐206 in U2OS cells. Furthermore, an inverse correlation between miR‐206 expression and ROR expression was observed in OS tissues. Importantly, down‐regulation of miR‐206 expression partially abrogated the functional effect of ROR knockdown on OS cell proliferation, colony formation, migration and invasion. These data provided reliable evidence suggesting that knockdown of ROR inhibited OS progression, at least in part, via regulation of miR‐206.

In conclusion, the present study showed that ROR expression was up‐regulated in OS tissues and cell lines, and associated with poor prognosis in OS patients. Furthermore, we demonstrated that knockdown of ROR significantly inhibited the proliferation, colony formation, migration and invasion of OS cells in vitro, as well as suppressed tumour growth in vivo by regulating miR‐206. Further studies are required to investigate its underlying mechanism for developing ROR as a potential therapeutic target for OS.

## CONFLICT OF INTEREST

The authors declare no conflict of interest.
